# An experimental study on stress-shielding effects of locked compression plates in fixing intact dog femur

This article has been retracted.

**DOI:** 10.1186/s13018-021-02238-3

**Published:** 2021-01-29

**Authors:** Xinwen Zhao, Wensen Jing, Zhe Yun, Xun Tong, Zhao Li, Jiajia Yu, Yaohui Zhang, Yabin Zhang, Zhixue Wang, Yanhua Wen, Heping Cai, Jun Wang, Baoan Ma, Haien Zhao

**Affiliations:** 1 Department of Joint Surgery, Yuncheng Hospital, The Eighth clinical Medical University, Shanxi province, 441000 China; 2 Department of Orthopedics, Honghui Hospital, Xi’an Jiaotong University, 555 Youyi East Road, Beilin District, Xi’an, 710054 Shaanxi Province China; 3 Department of Orthopedics, 941st Hospital of PLAJLSF, Xining, 810000 Qinghai proviince China; 4 Department of Traditional Chinese Medicine Rehabilitation and Physiotherapy, Xuzhou Army 71st Group Army Hospital, Xuzhou, 221000 Jiangsu province China; 5 Institution of Orthopedics, Tangdu Hospital, Air Force Medical University, Xi’an, 710038 Shaanxi province China; 6 School of Materials Science and Engineering, Xi’an Jiaotong University, Xi’an,710061 shaanxi province, China; 7 Center of Orthopedic laboratory, Xijing Hospital, Air Force Medical University, Xi’an, 710038 Shaanxi province China

**Keywords:** Stress-shielding effects, Osteopenia, Osteoporosis, MIPPO technique, Plate fixation, LCP, LC-DCP

## Abstract

**Background:**

In orthopedic application, stress-shielding effects of implant materials cause bone loss, which often induces porosis, delayed bone healing, and other complications. We aimed to compare the stress-shielding effects of locked compression plate (LCP) and limited-contact dynamic compression plate (LC-DCP) in dogs with plate-fixed femurs.

**Methods:**

Bilateral intact femurs of 24 adult dogs were fixed by adult forearm 9-hole titanium plates using minimally invasive plate osteosynthesis (MIPPO) technology, with LCP on the left and LC-DCP on the right femurs. Dogs were sacrificed at 6 weeks, 12 weeks, and 24 weeks after surgery, and bone specimens were used to evaluate the efficacies of different fixing methods on bones through X-ray, dual-energy X-ray absorptiometry (DEXA), histology, MicroCT, and biomechanics analyses.

**Results:**

X-ray results showed significant callus formation and periosteal reaction in the LC-DCP group. Bone cell morphology, degree of osteoporosis, and bone mineral density (BMD) changes of the LCP group were significantly better than that of the LC-DCP group. MicroCT results showed that the LCP group had significantly reduced degree of cortical bone osteoporosis than the LC-DCP group. Tissue mineral density (TMD) in the LCP group was higher than that in the LC-DCP group at different time points (6 weeks, 12 weeks, and 24 weeks). Biomechanics analyses demonstrated that the compressive strength and flexural strength of bones fixed by LCP were better than that by LC-DCP.

**Conclusions:**

Stress-shielding effects of LCP are significantly weaker than that of LC-DCP, which is beneficial to new bone formation and fracture healing, and LCP can be widely used in clinic for fracture fixation.

## Background

Plates for internal fixation of fractures have been used for more than 100 years [1]. Although initial shortcomings such as corrosion and insufficient strength have been overcome, better designs are still needed to develop a plate that accelerates fracture healing while not interfering with bone physiology [2]. Plate fixing intact femur may induce osteopenia and osteoporosis, and such adverse effects are becoming more and more the concerns for the patients [3]. Clinical studies and investigations with animal models have revealed that the degree of osteopenia and osteoporosis after femur plate fixation may be varied depending on different plates at different periods [2, 4, 5]. Based on previous studies in dogs [4, 6], plate fixing intact femur of dogs may result in two effects: short-term effect and long-term effect. The former includes the influence of blood supply of fixed bone in the early 8 weeks, while the latter mainly refers to the stress shielding effect, an effect of reduction in bone density as a result of removal of typical stress from the bone by an implant [7]. These two effects result in decreased bone mass and reduced bone strength due to plate fixation, both of which are independent as well as super-imposed. After certain time of about 8 weeks, effects of blood supply on bone vanish due to revascularization, with only stress-shielding effect left acting on bones fixed by plates, which may change the process and determine final formation of bones [7]. The production of these two effects are correlated with the contact area of plate and bone surface as well as the plate strengt h[8], but there has been no clear conclusion on degree changes of stress-shielding effect of bones fixed by plates so far.

Due to the developments in improving internal fixation materials and minimizing contact area between plate and bone surface, LCP (locked compression plate), as a locking internal fixator [9], has been successfully used in clinic for over one decade. It has the characteristics of minimum contact between the external fixator and the bone, as well as between the steel plate and the bone surface [10, 11]. Since it has reduced number of fixing force arm, the fixing strength of LCP is significantly enhanced. Coupled with its unique advantages in design, LCP can fulfill the use of minimally invasive percutaneous plate osteosynthesis (MIPPO) technology to achieve satisfactory fixation and reduce the chance of nail exposure-caused needle track infections [10, 11]. However, whether LCP leads to stress shielding effect of bones has not been extensively studied so far. LC-DCP (limited contact dynamic compression plate), as the name implies, is a limited-contact compression plate that is also widely used in clinic [1, 12]. The contact area of LC-DCP with the bone surface is relatively larger than that of LCP and the contact strength is tighter [12]. Since the damage to blood supply and transportation in LC-DCP fixed bones is relatively more severe than that in LCP fixed bones [12], it is presumably that the long-term stress shielding effect of LC-DCP could be more evident than that of LCP. However, this hypothesis lacks experimental supports.

Due to bioethics and legal issues, there is an applicable research method to investigate characteristics of implant materials using large animals with similar anatomical and mechanical properties, which has been described in the internationally universal 3 R humanitarian principle: Reduction, Refinement, Replacement [13, 14]. It was reported that LCP constructs were significantly more resistant to compression than LC-DCP constructs in an in vitro comparison in the femur of newborn calves [15]. In addition, monocortical LCP fixation was considered as a more effective treatment option than LC-DCP for nonunion of femur shaft fracture occurred after intramedullary nail fixation [16]. Moreover, in a canine femoral fracture-gap model, the LC-DCP with an intramedullary rod (LC-DCP-R) showed higher stiffness and resistance to failure, lower interfragmentary motion, and lower plate strain and stress compared to LCP [12]. Nevertheless, more intensive comparisons on the efficacy of the surgical treatments with LCP and LC-DCP, especially the long-term stress shielding effect, are required to provide better guidance for clinical therapy. In recent years, MicroCT (micro-computed tomography) has been applied to achieve accurate segmentation of images to better characterize the properties of cortical bone, trabecular bone, and newborn bone after plate fixation [15, 16]. In addition, the critical parameters derived from the MicroCT analyses, including tissue mineral density (TMD), trabecular thickness (Tb.Th), trabecular number (Tb.N), and trabecular separation (Tb.Sp), are considered to be able to more accurately reflect the degree of osteopenia and osteoporosis in quantities [17, 18]. Therefore, these advanced tools can be used to facilitate the investigations on the efficacy of plates used for bone fixing.

In the present study, a two-phase experiment was designed to compare the effects of LCP fixation and LC-DCP fixation on biological properties of bones in dogs with plate-fixed femurs. Through the use of tools like X-ray, histology, dual energy X-ray absorptiometry (DEXA), MicroCT combined with biomechanical testing, the morphological and histological appearances, as well as the biological and functional properties of bones after plate fixation for different periods were examined. On the first phase, we aimed to examine the short-term effects of plates on fixed bones at the time points of 6 weeks and 12 weeks, including the full periosteum formation under plates which required about 6 weeks, and the complete recovery of blood supply which required about 6–12 weeks. During 12–24 weeks, the stress-shielding effect was the only concern. Therefore, on the second phase, we focused on the long-term stress shielding effect and explored the possible functional changes of bones in dogs with LCP fixation and LC-DCP fixation of femurs for 24 weeks.

## Methods

### Animals

Twenty-four adult healthy mongrel dogs (random mix of male and female dogs, with age of 1.5–2.5 years old and body weight of 20 ± 5 kg as suitable for plate fixing) were provided from the Animal Center of The Air Force Medical University (Xi’an, China). The femur length of all the dogs was suitable for fixation by a 9-hole titanium plate. These dogs were divided into 3 time point groups (6-week, 12-week, and 24-week time point groups), with 8 dogs each time point group and 4 dogs in LCP or LC-DCP group for each time point. Dogs were housed at the specific pathogen-free (SPF) facility at the Animal Center of The Air Force Medical University at room temperature (22 ± 1 °C) with a 12/12 h light/dark cycle and access to food and water ad libitum. All animal experiments involving the use of dog in this study were approved by the Institutional Animal Care and Use Committee of Hospital.

### Plate fixing of dog femurs

Xylazine hydrochloride injection at the dose of 3.2 mg/kg and combined with propofol injection at the dose of 2.0 mg/kg body weight was used for intramuscular anesthesia. LCP (adult forearm 9-hole titanium plate, Kanghui, China) was fixed on left femur using the minimally invasive percutaneous plate osteosynthesis (MIPPO). Three locking screws were inserted on 134 screw holes (middle screw holes as boundary) of both sides of the plate (6 screws in total). Incision was sutured layer by layer after saline flush. LC-DCP (adult forearm 9-hole titanium plate, Kanghui, China) was fixed on right femur using the same method as LCP. Penicillin of 1.6 million units was intramuscularly injected both preoperatively and postoperatively on surgery day. The first day after surgery, penicillin of 1.6 million units was intramuscularly injected twice to reduce risk of post-operative infection. The surgeries were grouped and managed respectively.

### Post-operative X-ray and specimen preparation

Post-operative X-ray review on bilateral femurs was performed on 1 week after surgery, and specimens were obtained to observe changes in femurs. Epilation and skin preparation on surgical area of bilateral femurs of dogs were performed on 1–2 days prior to surgery, followed with routine dual-energy X-ray absorptiometry (DEXA). Eight dogs were sacrificed on 6 weeks, 12 weeks, and 24 weeks post-operation, respectively, and plates were removed for DEXA to generally observe histological conditions and callus formation around bones fixed by plates. The bilateral femurs were obtained with removing soft tissues and amputating upper and lower joint to maintain bones fixed by plates as specimens, which were further processed to appropriate size in accordance with experimental requirements.

### DEXA tests

DEXA analyzer (IDAX, GE Healthcare, Wauwatosa WI, USA) from Radiology Department of Hospital was adopted to perform preoperative and postoperative DEXA tests on dogs at different time points. The preoperative and postoperative BMD differences from the same group at the same time point were compared by performing paired *t* test.

### Histological observation

Specimens adopted methyl methacrylate (Damao Chemical Reagent Factory, Tianjin, China) to perform undecalcified plastic embedding, and LeikaSP1600 hard tissue slicer (Frankfurt, Germany) was used to obtain slices of 50 μm. After staining of Ponceau trichrome (ShangHai SSS Reagent Co., Ltd), histological observation was performed under an optical microscope, with all images enlarged by 40 times for analysis.

### MicroCT three-dimensional imaging analysis

Bone specimens obtained from 6-week, 12-week, and 24-week time point group were cut to the appropriate size (length of 2 cm). A group of two specimens at the same time point with one from the LCP group and one from the LC-DCP group were vertically placed in a scanning tube, and then the tube was placed on GE eXplore Locus SP Micro-CT from Institute of Orthopedics of Hospital for scanning with a scanning time of around 210 min. Original mini-vol files acquired from the scanning were opened to perform accurate three-dimensional reconstruction of all images and data analyses using Micview V2.1.2 three-dimensional reconstruction processing software (GE Healthcare). Using 0.5 cm as a length unit, each specimen was equally divided into 4 bone segments in combination with ABA special bone analysis software (GE Healthcare) to obtain TMD value of each scanned bone segment. The results above were used to perform paired *t* test to compare if there were significant differences for both plate fixations in osteoporosis degree of corresponding bone segments at different periods.

### Biomechanical analysis

Femoral specimens fixed by plates at different periods were processed into samples with a length of 11 cm or 3 cm. The INSTRON Mechanical testing machine (Instron, Canton, UK) from the Institute of Materials and Strength of Xi’an Jiaotong University was used for three-point bending test (11 cm specimens, with carrier spacing of 7 cm) and compression test (3 cm specimens). Data of average flexural strength values or compressive strength values were collected and calculated.

### Flexural strength and compressive strength

Flexural strength and compressive strength of bones are important indicators for bone mechanics. Flexural strength means unit area load value when loading between two points of specimen until it is broken. The formula is from “YBT 5349-2006 metal bending mechanical performance testing method,” as is ${\sigma}_{bb}=\frac{F_{bb}\times {L}_s}{4W}$, round bar specimen: $W=\frac{\pi {d}^3}{32}$ to get ${\sigma}_{bb}=\frac{8\times {F}_{bb}\times {L}_s}{\pi {d}^3}$ (*σ*_*bb*_ - flexural strength/MPa, *F*_*bb*_ - maximum bending load/kN, *L*_*s*_ - span/mm; *d*—diameter of round bar specimen/mm).

Compressive strength, known as σbc, is the strength limit of pressure. Because *σ*_*bc*_ is reversely correlated with *S*_0_, maximum tensile strength is calculated by the minimum cross-sectional area, and average compressive strength is calculated by the average cross-sectional area. The formula is ${\sigma}_{bc}=\frac{F_{bc}}{S_0}$ ${S}_0=\frac{\pi {d}^2}{4}$ (*σ*_*bc*_—tensile strength/MPa; *F*_*bc*_—the maximum compression force /*N*; *S*_0_—original cross-sectional area/mm^2^; *d*—average diameter of specimen).

### Statistical analysis

Statistical analysis was performed using SPSS 16.0 software (SPSS, Inc., Chicago, IL, USA). Data in each figure represent the mean ± standard deviation (S.D.) from at least three independent experiments. Differences between the two groups were compared using the two-tailed Student's *t* test and one-way analysis of variance (ANOVA). A *P* value less than 0.05 was considered statistically significant.

## Results

### Postoperative X-ray results demonstrate better morphological bone recovery in LCP-fixed dog femurs

LCP and LC-DCP were fixed on the left femur and right femur of dogs, respectively, using the MIPPO technology (Fig. 1), and the post-operative effects of bone fixation with these two plate approaches were observed and compared at 6 weeks, 12 weeks, and 24 weeks after surgery. Post-operative activities of dogs were observed with bilateral femurs as self-controls. The results of postoperative X-ray showed that bilateral femurs were fixed in good position for both plates (Fig. 2a, b), with no significant cyst formation (Fig. 2c, d). After plates were removed, X-ray results demonstrated that different bone reaction of bilateral femurs fixed by plates, which was more significant for LC-DCP group in callus formation and periosteal reaction (Fig. 2e, f). Density of bones around screw channel of LC-DCP group was slightly lower than that of LCP group (Fig. 2g, h). Therefore, morphological bone recovery in LCP-fixed dog femur was better than that in LC-DCP-fixed dog femur.

**Fig. 1:** Representative images show the processes of fixation of dog intact femur with LCP and LC-DCP by the MIPPO technology. **a**, **b** The pictures of 9 holes locking plate (LCP, **a**) and 9 holes limiting contact dynamic compression plate (LC-DCP, **b**). **c**, **d** The pictures show the insertion of LCP in dog left femur (**c**) and LC-DCP in dog right femur (**d**) by MIPPO. **e**, **f** The pictures show the fixation of LCP in dog left femur (**e**) and LC-DCP in dog right femur (**f**) by screws

**Fig. 2:** Comparison of the morphological bone recovery in LCP and LC-DCP fixed dog femurs by postoperative X-ray assays. **a**–**h** Representative images show the position of bilateral femurs (**a** and **e**; LCP on left, and LC-DCP on right), the callus formation of bilateral plates (**b** and **f**; LCP on left, and LC-DCP on right), bone formation around screw channel (**c** and **g** for LCP; **d** and **h** for LC-DCP) at 12 weeks (**a**–**d**) and 24 weeks (**e**–**h**) after surgery. **i** The descent value of DEXA at different time points (6 weeks, 12 weeks, and 24 weeks) for the LCP and LC-DCP plates were summarized. *n* = 4 for each group; *P < 0.05, compared with the LCP group

### DEXA tests revealed that LCP-fixed dog femurs displayed lower decrease degree of bone mineral density (BMD) than LC-DCP-fixed dog femur

We also performed statistical analyses on descent value of DEXA at different periods for both plates. The results revealed that the decrease degree of BMD gradually increased from 6 weeks to 12 weeks. The decrease degree of BMD in the LCP group was lower than that in the LC-DCP group at the same time points, while significant difference in the descent value of DEXA was observed at each period (*P* < 0.05). When fixation time prolonged to 24 weeks, the decrease degree of BMD was gradually reduced, especially for that of the LCP group (Fig. 2i). Thus, LCP-fixed dog femur was less tended to have bone loss than the LC-DCP-fixed dog femur.

### The LCP group had better histological conditions of bones than the LC-DCP group

We conducted hard tissue sections with Ponceau trichrome staining to further examine the histology of bones after plate-fixation. It can be concluded from images of 6-week hard tissue section staining that the bone area of the LCP group was bigger than that of the LC-DCP group, with better bone mineralization and less osteoporosis degree for LCP group (Fig. 3a, d). At 12 weeks after surgery, the cortical bone morphology of the LCP group was nearly normal with better bone mineralization while the LC-DCP group demonstrated signs of osteoporosis (Fig. 3b, e). Osteoporosis of the LC-DCP group at 24 weeks was significantly more aggravated than that of 12 weeks, whereas osteoporosis of the LCP group was only slightly increased. In addition, bone density of the LCP group at 24 weeks was significantly higher than that of the LC-DCP group (Fig. 3c, f). Collectively, histological conditions of bones in the LCP group were better than that in the LC-DCP group at each examined time point.

**Fig. 3:** Comparison of the histological conditions of bones fixed by LCP and LC-DCP for different periods. **a**–**f** The histological conditions of bones were examined by staining with Ponceau trichrome. Representative images show the staining results for the bones fixed by LCP (**d**–**f**) and LC-DCP (**a**–**c**) at 6 weeks (**a**, **d**), 12 weeks (**b**, **e**), and 24 weeks (**c**, **f**) after surgery. Magnification, × 40

### MicroCT tests revealed that LCP resulted in lower degree of osteoporosis and osteopenia than LC-DCP

To further quantitate the osteoporosis and osteopenia degree, we employed MicroCT tests to determine the morphological changes of cortical bone (Fig. 4) and newborn bone of screw channel of the corresponding bone segments (Fig. 5) fixed by two plates at different periods. While 6-week fixation resulted in no significant osteoporosis of the cortical bone, which was basically as close as the normal cortical bone (Fig. 4a, d), 12-week fixation resulted in the most serious osteoporosis degree of cortical bone, especially for the LC-DCP group (Fig. 4b, e). When fixation time prolonged to 12 weeks, osteopenia degree increased significantly, especially for the LC-DCP group (Fig. 4b, e). When fixation time prolonged to 24 weeks, osteopenia degree was improved significantly, with cortical bone getting dense and thickness of cortical bone increased (Fig. 4c, f), and the TMD value corresponding with the image was also elevated significantly, especially for the LCP group (Fig. 4g). Similar trends on the morphological changes of newborn bone of screw channels were noticed. The Tb.Th and Tb.N values of newborn bone around screw channels for the LCP group increased significantly and the Tb.SP value decreased significantly (Fig. 5), indicating the strength of newborn bone was gradually increasing. Notably, the strength of newborn bone in the LCP group was better than that of the LC-DCP group at all time points except on 6-week fixation (Fig. 5). Taken together, these MicroCT results suggest that the stress-shielding effect of LCP on fixed bone segment was significantly lower than that of LC-DCP.

**Fig. 4:** The morphological changes of cortical bones fixed by LCP and LC-DCP for different periods were examined by MicroCT. **a**–**f** Representative images show the morphology of the cortical bone around one screw at different periods (6 weeks, **a** and **d**; 12 weeks, **b** and **e**; 24 weeks, **c** and **f**) for different plates (LC-DCP, **a**–**c**; LCP, **d**–**f**). The parameters were as follows: height of 5 mm, threshold of 1800; ROI completely included the lateral cortical bone; and the cortical bone was displayed as the pseudo color brown for distinction. **g** The TMD values at different time points (6 weeks, 12 weeks, and 24 weeks) for the LCP and LC-DCP plates were summarized. *n* = 4 for each group; *P < 0.05, **P < 0.01, compared with the LCP group

**Fig. 5:** The morphological changes of newborn bone around the screw channel in the LCP and LC-DCP groups for different periods were examined by MicroCT. **a**–**f** Representative images show the morphology of the newborn bone around the screw channel at different periods (6 weeks, **a** and **d**; 12 weeks, **b** and **e**; 24 weeks, **c** and **f**) for different plates (LC-DCP, **a**–**c**; LCP, **d**–**f**). The parameters were as follows: height of 5 mm, threshold of 600, with pith; intramedullary normal bones were completely removed to prevent influence on images; and the newborn bone was displayed as the pseudo color blue for distinction

### The mechanical properties of bones fixed by LCP were superior to that of bones fixed by LC-DCP

To compare the mechanical properties of bones fixed by LCP and LC-DCP, we performed biomechanical testing to determine the compressive strength and flexural strength of bones harvested at different time points. We found that the average compressive strength in both LCP and LC-DCP groups decreased on 12-week fixation, and the compressive strength of the LC-DCP group reached the highest level on 24-week. However, the compressive strength of the LCP group was always better than that of the LC-DCP group at the same time point, and there were significant differences between the values of these two groups (*P* < 0.05; Fig. 6a). For each group, there were no significant changes for the average flexural strength between 6 weeks and 12 weeks. However, there were significant differences between the LCP group and the LC-DCP group at each time point (*P* < 0.05; Fig. 6b), indicating that the flexural strength of LCP was superior to that of LC-DCP at the same period after surgery. Therefore, the mechanical properties of bones fixed by LCP were superior to that of bones fixed by LC-DCP.

**Fig. 6:** Comparison of the compressive strength and flexural strength of bones fixed by LCP and LC-DCP for different periods. **a**, **b** The compressive strength (**a**) and flexural strength (**b**) of bones at different time points (6 weeks, 12 weeks, and 24 weeks) after fixation with the LCP and LC-DCP plates were summarized. *n* = 4 for each group; *P < 0.05, compared with the LCP group

## Discussion

Plate fixing of femur can lead to both short-term effect, which influences blood supply of fixed bone area, and long-term effect, which results in decreased bone mass and reduced bone strength [1, 2]. Productions of the two effects are correlated with the contact area of plate and bone surface as well as plate strength [8, 9, 19, 20]. However, there is no intensive study on elucidating the differences in the impacts of two widely used plates, LCP and LC-DCP, on the short-term and long-term effects of bones fixed by plates. In this study, we established an animal model of plate-fixed intact femur in dogs and evaluated the morphological and histological changes, as well as the biological and functional properties of the bone area of dogs bearing LCP and LC-DCP fixed femurs for 6 weeks, 12 weeks, and 24 weeks. Our results demonstrated that LCP was superior to LC-DCP in terms of morphological bone recovery, decreasing the degree of bone mineral density, histological conditions, degree of osteoporosis and osteopenia, and biomechanical properties of fixed bone area.

Axial pressing action of screw between traditional plate and bone surface often results in close contact between the plate and bone surface, which produces huge frictional force to maintain the stability for fixation. Therefore, artery blood supply and venous reflux disorder of cortical bone were induced [21]. In 1974, Rhinelande et al. reported that there was indeed cortical bone ischemia under the plate, where it was along the screw centerline, and only a very narrow longitudinal area, and capillaries may be easily distributed below the edge of the plate in this area [22]. Gunst et al. found cortical bone ischemia occurred 10 min after surgery when complete tibiae of rabbits were fixed by plates [23]. After 24 h, cortical bone ischemia was further aggravated and affected surrounding whole layer of the cortical bone below the plate. Ischemia area was reduced after 3–4 weeks, and blood supply of most area was recovered in 8–12 weeks [23]. Perren et al^.^ found that plates may significantly interfere with blood supply of cortical bone through using the in vivo dye diisobutylthiuram disulfide as markers [24]. In addition, mechanical bone mass loss due to stress shielding and impaired blood perfusion of cortical bone resulting from wide contact between bone and plate may induce necrosis of cortical bone [1, 11]. Therefore, based on the above known knowledge, it is urgent to innovate the design of plates used for femur fixing to avoid the side effects like cortical porosis, delayed bridging, and refractures after plate removal. Due to bioethics and legal issues, it is impossible to directly conduct implant experiments in humans. Instead, an applicable research method to investigate characteristics of implant materials is using large animals with anatomical and mechanical properties similar to humans. The clinical effects of implant materials observed in these animals can be extended to humans. Such a research method has been internationally recognized and universally practiced, as well as described in the internationally universal 3 R humanitarian principle [13, 14]. Commonly used animals for mechanical properties of implant materials include dogs, sheep, cows, and pigs, which are available at low-cost but easy to manage. In this study, hind limbs of dogs were chosen for studying the stress-shielding effect under plate-fixing. Hind limbs of dogs have similar anatomical characteristics with those of humans, with operation reality and availability. Moreover, like the lower limbs of humans which function for walking upright, the hind limbs of dogs are also responsible for weight-bearing support. This models a similar role in humans and thus the effect of plate fixation on dog’s femur can be extended to humans and used for clinical promotion. In addition, the effect of plate fixation is not limited by the size of the plate and can be extended to different populations and positions of humans. Therefore, the experimental results of animals are also applicable to the plate fixation of long tubular bones of humans.

Changes in blood supply and stress-shielding effect are main consequences deriving from plate-fixing and correlated with the contact area of plate and bone surface as well as the plate strength [8]. There are several reasons that we have selected the intact femur as the model for stress-shielding effects of LCP and LC-DCP. On one hand, it is technically impossible to generate fractures that are identical across the animal individuals in the experiment. Factors such as distance between fracture ends, location and type of the fracture, internal fixation strength, distance between fixation screws and fracture ends, and the length of the fixation nail could all vary. The variations are easy to perturb the accuracy of results. Therefore, it is unlikely to study the stress-shielding effect alone in a fracture model. On the other hand, blood supply is an important factor affecting fracture healing; however, changes in blood supply as a result of plate-fixing will likely differ because of nutrition status and internal fixation status. Therefore, individual differences of the recovery time for weight-load walking could be significant. In addition, bilateral femoral shaft fracture modeling may cause higher risk of postoperative infection and mortality, leading to paired samples uneasy to be achieved in the experiment. As stated above, using a fracture model may bring more uncertainty to the results which may become inaccurate or even invalid. In contrast, using an intact femur model allows an early recovery for weight-load walking and avoids the occurrence of atrophy and osteoporosis caused by prolonged immobilization after surgery, thereby minimizing the effect of interference factors on the stress shielding effect of the steel plate influences. Furthermore, LCP is independent on friction between bone and plate, and satisfactory fixation is achieved through no contact of bone surface. Therefore, early temporary osteoporosis, the common disadvantage of traditional plates, can be avoided [25]. As the development and wide clinical application of LCP, as well as deeper research on biomechanical properties of LCP, there are new findings and advancements for LCP in biomechanics [26]. Meanwhile, some investigators studied stress-shielding effects of LCP under simulated ideal conditions (not considering effects of blood supply on fixed bones) through finite element analysis and concluded that LCP may better maintain stability of fixation and reduce stress-shielding effect of plates [27]. These are the unparalleled advantages that were not found in traditional plates. In this study, for taking blood supply into account to objectively and realistically reflect the stress-shielding effect of LCP, we designed a two-phase experiment and used LC-DCP as a control group. In addition, the bilateral intact femurs of one dog can be considered as self-control group, and LCP and LC-DCP were used in the same dogs, which could minimize the effects of other factors other than the plates.

On the first phase, morphological and histological appearances of bones fixed by different plates for different periods were observed to confirm that full periosteum formation under plates required about 6 weeks, and complete recovery of blood supply required about 6–12 weeks. These were the demonstrations of the namely short-term effects of plates on fixed bones (as well as effects on blood supply). After 12–24 weeks, only stress-shielding effect remained as the concern, as previously reported [28]. The results demonstrated that periosteum formation process for the LC-DCP group was from scratch, and it was periosteum re-shaping process for the LCP group. There was new periosteum formation for both the LCP and LC-DCP groups on the time point of 6 weeks and completely normal periosteum form after 12 weeks we observed in both groups, which was basically consistent with study from Uhthoff, H.K [4], namely the synergistic time needed for emerging the effects on blood supply and stress-shielding effects in plate-fixed intact femurs was around 8 weeks [4]. However, we demonstrated that periosteum formation of bones fixed by plates was basically completed after 6 weeks in an intuitive way, and complete blood supply recovery required no more than 12 weeks. On the second phase, stress-shielding effect of LCP on bones was scientifically and accurately reflected, and all results comprehensively revealed that the stress-shielding effect of LCP was significantly lower than that of LC-DCP.

Results of hard tissue sections with Ponceau trichrome staining revealed that osteoporosis degree of the LC-DCP group increased significantly from 6 weeks to 24 weeks, and osteoporosis degree reached the peak at 24 weeks. However, osteoporosis degree in the LCP group basically remained almost the same at three time points, with just a very slightly increasing tendency. Histological conditions of bone at corresponding periods were all better in the LCP group than the LC-DCP group. Between 6 weeks and 12 weeks after fixation, the bone changes of the LC-DCP group may be correlated with reactive stimulation due to local ischemic disorders caused by early plate fixation compression. When fixation time prolonged to 24 weeks, the cortical osteoporosis in the LC-DCP was further more aggravated comparing to that of 12 weeks. During this period, owing to the blood supply of bone fixed by plates being basically recovered, the aggravation of osteoporosis degree was positively correlated with stress-shielding effect of LC-DCP. As for the LCP group, from 6 weeks to 24 weeks, because there was no close contact between LCP and bone surface, early temporary osteoporosis due to local ischemic disorders was avoided. When fixation time prolonged to 24 weeks, single action of stress-shielding effect may lead to a very slightly increased osteoporosis degree. However, the overall stress-shielding effect of LCP at this time point was significantly weak than that of LC-DCP. For example, from the results of MicroCT tests in terms of images or TMD data demonstrating characters at different periods, we can conclude that the osteoporosis degree in the LCP group was less than that in the LC-DCP group, even as the fixation time prolonged, indicating that stress-shielding effects of LCP on bones were significantly weaker than that of LC-DCP, which was beneficial to callus and newborn bone formation.

## Conclusion and prospects

The results of this study were obtained from intact femur fixation, which was quite different from clinical fracture. Although properties and stress-shielding effect of LCP was reflected to a certain degree, especially with emphasizing on its advantages comparing to LC-DCP, the fracture healing effects of LCP require further demonstrations under realistic fracture fixation conditions. Meanwhile, whether stress-shielding effect of plate fixation exists for a long time and the specific correlation between the action of LCP and prolong of fixing time are still unknown. As revealed by histological section image and MicroCT, contralateral bone form differences under fixations with different plates may indicate the disadvantage of LCP-mediated femur fixation at early time points. However, considering the significantly reduced stress-shielding effect in dog experiments, LCP might be superior to LC-DCP in plate fixation of femur fractures.

## Data Availability

Data sharing is not available.

## Abbreviations

LCP: Locked compression plate
LC-DCP: Limited-contact dynamic compression plate
MIPPO: Minimally invasive plate osteosynthesis
DEXA: Dual-energy X-ray absorptiometry
BMD: Bone mineral density
TMD: Tissue mineral density
LC-DCP-R: LC-DCP with an intramedullary rod
Tb.Th: Trabecular thickness
Tb.N: Trabecular number
Tb.Sp: Trabecular separation
